The article "Real-Time Detection of Body Nutrition in Sports Training Based on Cloud Computing and Somatosensory Network" was retracted in 2023. Reasons: signs of a paper mill; suspected computer-generated content; unreliable results or conclusions; concerns about the data.

# Real-Time Detection of Body Nutrition in Sports Training Based on Cloud Computing and Somatosensory Network

**DOI:** 10.1155/2022/9911905

**Published:** 2022-04-15

**Authors:** Ruyao Gong, Nan Ge, Jijie Li

**Affiliations:** ^1^College of Sports and Health, Linyi University, Linyi 276000, Shandong, China; ^2^Physical Education, Kunsan National University, Gunsan 54150, Jeollabuk-do, Republic of Korea

## Abstract

With the progress of society and the improvement of living standards, sports training has gradually become an area of increasing concern for society and individuals. To more comprehensively grasp the physical function, body shape, and physical fitness of athletes, many researchers have conducted extensive research on the real-time detection of human body nutrition. This study is mainly supported by cloud computing and somatosensory network technology, and the real-time detection of human body composition in sports training is the main research object. In the experiment, two methods of human body composition detection were tested: the BIA method and the body composition analysis method based on the electrochemical sensor of body sweat. It designed a human nutrient composition detection system based on the BIA method. The error rate of the system is relatively small, which is basically maintained at about 2%. It uses a body surface sweat electrochemical sensor to detect changes in glucose concentration during human exercise. After exercising for a period of time, the test subject's sweat glucose concentration remained around 0.5 mM.

## 1. Introduction

Sports training is the repetitive work of systematically carrying out similar physical or mental activities. It can cause an adaptation process in the body, leading to the maintenance or enhancement of exercise capacity. In this process, it is necessary to control the body's nutrition to maintain a certain level; otherwise, the balance between exercise fatigue and exercise recovery will not be reached. Therefore, it is necessary to conduct real-time detection of body nutrition during sports training. And the rapid development of chip technology and wireless communication technology has made it possible.

Due to the use of wireless transmission, easy access to data, small node size, and low cost, human sensor networks have broad potential in fields such as healthcare, biomedicine, and physical training. The digital development and miniaturization of sensors help to gradually apply human sensor network applications to people's daily lives. This technology has developed very rapidly in recent years, and the technology contained in the sensor will not cause any inconvenience. However, in some application areas, such as monitoring human health and determining behavior, there are relatively high requirements for real-time data availability and collection frequency; therefore, further research is needed. The massive data processing technology of cloud computing technology can ensure that the underlying user's physical data is accurately and securely connected to the system, thereby ensuring the accuracy of the processing results. Cloud computing greatly improves the efficiency of data processing, making the entire platform more efficient.

The human body composition analysis system based on cloud computing and somatosensory network can effectively and better serve sports trainers and the general public. Data analysis of their physical health status, an evaluation report, and real-time return to the server through the cloud platform can help users arrange fitness exercises and predict their physical condition more rationally and scientifically.

## 2. Related Work

Zhenni studied the real-time dynamic changes of hypochlorite and ascorbic acid in the human body. He proposed a nanosensor with good fluorescent probe performance. It can be used for the dynamic detection of hypochlorite and ascorbic acid in living cells, which can be monitored by fluorescence microscopy [1]. His research and development have certain reference significance for real-time detection of human body health, but the performance of the nanosensor he proposed needs to be further improved. The purpose of Bagnaka's research is to expand the previous research by using machine learning models to explore the classification of fNIRS signals (oxyhemoglobin) based on temperature levels (cold and hot) and corresponding pain intensity (low and high). However, his research field is slightly different from this study on physical nutrition testing in sports training, which may not have many references. Ribeiro proposed a decision-making method to help decision makers determine their priorities in the process of selecting system projects compatible with cloud computing technology. The method is based on the AHP method, and the hierarchical structure is composed of multidisciplinary standards, with a total of four standard categories and 20 substandards [2]. However, his research method is too complicated and requires a lot of resources. Fog computing introduces an intermediate layer of fog between mobile users and the cloud and supplements' cloud computing for low-latency and high-speed services for mobile users. Deng studied the trade-off between power consumption and transmission delay in the fog cloud computing system and proposed a workload distribution problem. This problem suggests that, under the condition of limited-service delay, the optimal workload distribution between fog and cloud is with minimum power consumption [3]. Any organization trying to achieve the best flexibility and quick response to market requests can choose to use cloud services. Chang provides a neutral multicriteria decision analysis (NMCDA) method to evaluate the quality of cloud services, thereby helping decision makers evaluate different cloud services. The triangular neutron number is used to deal with the fuzzy and incompatible information that usually exists in PE [4]. Hirai considers the efficiency of backup tasks in cloud computing. He modeled the task scheduling server as a single server queue, where the server is composed of multiple workers. When the task enters the server, the task is split into subtasks, and each subtask is served by its own auxiliary task and another different auxiliary task [5]. Wennberg tried to determine whether a magnetoencephalogram (MEG) could reliably record the presence of neurophysiological dysfunction after an acute concussion. Based on previous studies of evoked potentials, he analyzed the somatosensory evoked field (SEF) caused by stimulating the median nerve of the wrist. He also designed case-control studies, established academic tertiary care centers, and assessed independent variables of risk factors [6].

## 3. Real-Time Detection of Body Nutrition in Sports Training Based on Cloud Computing and Somatosensory Network

### 3.1. Cloud Computing Technology

#### 3.1.1. Introduction to Cloud Computing

Cloud computing connects a large number of computer clusters with interconnection technology through hardware and software technology. It also combines operating modes with a powerful computer and online storage capabilities. Its main function is to realize distributed computing of a large amounts of data, parallel computing of large number of processes, storage of large network data, virtual shared network resources, resource configuration, load balancing, and storage of redundant data through hot backup [7, 8]. Users access the data center through mobile phone stations (such as computers, laptops, and mobile phones). It can customize the corresponding services as needed and can easily share unlimited applications and services provided by a large number of devices. Compared with traditional application platforms, cloud computing platforms have strong computing power, unlimited storage capacity, convenient and fast virtual services, cheaper cross-platforms, and high-cost performance. The cloud computing model architecture is shown in Figure 1.

#### 3.1.2. Cloud Computing Characteristics and Logical Structure

Cloud computing is different from traditional network computing and distributed computing. The difference is that cloud computing provides diversified services for multiple users, while grid computing services are single and special; cloud computing emphasizes that users have independent resource spaces, while grid computing shares resources. As shown in Figure 2, cloud computing completely combines business and technology, leading to the characteristics of cloud computing [9–11]. The first function is virtual, which summarizes the physical resource infrastructure and can arrange resources appropriately. The second function is multitenant, ensuring that users will not be disturbed. The third function is an on-demand service, where cloud providers charge fees based on user usage. The fourth function is scalability, which allows computer nodes to join or exit the server block at any time.

In the cloud computing structure, cloud users can choose service items according to their needs after obtaining the corresponding authorization through the cloud platform and requesting or canceling subscriptions. The cloud user decides the required service, and the management system is responsible for processing the user's request. System management allocates resources reasonably based on load balancing configuration, order distribution, and application configuration of deployment tools. The logical structure of cloud computing is shown in Figure 3.

#### 3.1.3. Cloud Computing Task Allocation

The cloud computing resource management model is divided into the application layer, connection layer, scheduling layer, and physical layer. Among them, the scheduling layer allocates resources according to different tasks and schedules the corresponding virtual machines. It ensures that the maximum performance of the physical server can be exerted as much as possible so that resources can be used to maximize the efficiency of the group. In cloud computing, the most widely used programming model is the Google Map/Reduce model. It consists of two parts. The first part is to divide the original task provided by the user into multiple subtasks, and the second part is to allocate each subtask to virtual resources. In the cloud environment, mutually independent subtasks are allocated to B virtual resource nodes for execution. Then, the task set is represented by formula (1) and the virtual resource node set is represented by formula (2):

(1) $$\begin{array}{c} W=\left\{w_{1},w_{2},\ldots ,w_{A}\right\}, \end{array}$$

(2) $$\begin{array}{c} V=\left\{v_{1},v_{2},\ldots ,v_{B}\right\}, \end{array}$$

where *w*_*i*_ represents the *i*th subtask and *v*_*j*_ represents the *j*th virtual resource, and each subtask can only be executed on one virtual resource. The assignment relationship between task set *W* and task set *V* can be represented by matrix *Z*:

(3) $$\begin{array}{c} Z=\left[\begin{array}{ccc} z_{11} & \cdots & z_{1A}\\ \vdots & \ddots & \vdots \\ z_{B1} & \cdots & z_{\text{BA}} \end{array}\right],\\ \sum_{j=1}^{B}z_{\text{ij}}=1,\;i\in \left(1,2,\ldots ,B\right),\;j\in \left(1,2,\ldots ,A\right),\\ \left\{\begin{array}{c} z_{\text{ij}}=1,\;\mathrm{if}\;w_{i}\text{ runs on }v_{j},\\ z_{\text{ij}}=0,w_{i}\text{ is not running on }v_{j}. \end{array}\right.. \end{array}$$

It is assumed that the characteristics of a cloud computing resource *C* can be expressed as

(4) $$\begin{array}{c} C_{i}=\left\{c_{i1},c_{i2},c_{i3},c_{iA}\right\}\;A\in \left[1,4\right]. \end{array}$$

Among them, *c*_*iA*_ represents the K-dimensional diagonal matrix and *c*_*i*1_, *c*_*i*2_, *c*_*i*3_, and *c*_*i*4_, respectively, represent memory, storage, CPU, and bandwidth.

The characteristics of the *i*-type task are

(5) $$\begin{array}{c} D_{i}=\left\{d_{i1},d_{i2},d_{i3},d_{iA}\right\}\;A\in \left[1,4\right];\sum_{j=1}^{B}d_{ij}=1. \end{array}$$

The following parameters need to be considered in the process of solving the optimization: network bandwidth band (*d*); network delay (*d*); and expected execution time *T* (*d*). Let *T*_*ij*_ be the expected execution time of the subtask *w*_*ij*_ in the virtual resource *v*_*Bi*_, corresponding to the matrix *Z*; then, the *T* matrix can be formed:

(6) $$\begin{array}{c} T=\left[\begin{array}{ccc} T_{11} & \cdots & T_{1A}\\ \vdots & \ddots & \vdots \\ T_{B1} & \cdots & T_{BA} \end{array}\right]. \end{array}$$

For network bandwidth and network delay, there are

(7) $$\begin{array}{c} \mathrm{Res}\;\left(d\right)=\frac{w_{1}T\left(d\right)+w_{2}\text{ delay}\left(d\right)}{w_{3}\text{ band}\left(d\right)},\\ \text{s}.\text{t}.\left\{\begin{array}{c} T\left(d\right)<\text{TL}\\ \text{band}\left(d\right)>\text{EL}\\ \mathrm{delay}\;\left(d\right)<\text{TL} \end{array}\right\}. \end{array}$$

The process of determining the optimal solution is the process of seeking the minimum Res (*d*), and *w*_1_, *w*_2_, and *w*_3_ are the weights of constraints, and TL, EL, and DL are boundary constraints.

### 3.2. Related Principles of Somatosensory Network

#### 3.2.1. Somatosensory Network

A wireless sensor network (WSN) is an intelligent system that monitors environmental variables with the help of a large number of deployed sensor elements. The working principles are as follows: a large number of sensor nodes are randomly distributed in a certain range of the target area, the data parameters in the area are collected according to specific needs, and the collected data are sent to the sink node in a single-hop or multihop communication mode. It then passes through the satellite connected to the console, and the user can search for data at the console and other terminals or issue “commands” to each node in the network. Its network structure is shown in Figure 4. The system structure is composed of sensor nodes, sink nodes, Internet, satellites, and consoles. The sensor node can be regarded as a kind of microembedded system, capable of data collection and fusion. It also needs to relay the data to other nodes [12–14].

Common routing protocols for wireless sensor networks include single-hop routing and multihop routing. They all have a common problem, that is, the system energy is not uniform. When using a single-hop routing model, nodes are far away from the base station. Due to the longer transmission distance, the energy consumption is faster, and when the multihop routing model is used, the nodes close to the base station forward a large amount of data, so the energy consumption is faster. Therefore, if any of them is used alone, the problem of uneven network energy consumption will occur, which will reduce the life of the system. To extend the life of the network, this study mainly introduces an improved routing protocol model. It is a hybrid routing protocol based on time components that combines the advantages of single-hop routing and multihop routing. Its structure is shown in Figure 5.

The energy consumption of the node transmitting the data packet to *p* is

(8) $$\begin{array}{c} {\text{EC}}_{T}={\text{EC}}_{\text{tr}}+\tau e^{\sigma }, \end{array}$$

where *τ* is the power amplification parameter, the energy consumption of the transmission circuit is represented by EC_tr_, *τe*^*σ*^ is the energy consumption to compensate the channel attenuation, and *σ* is the channel attenuation coefficient.

The network calculates its life cycle in rounds. A single-hop routing protocol is used for round *aT*, a multihop mode is used for (1 − *a*) *T*, and the value of *a* is greater than 0 and less than 1. When the *R*th layer node passes through the *aT* round, the average energy consumption is

(9) $$\begin{array}{c} {\text{EC}}_{1}\left(\text{Rw}\right)=\text{aT}\left[A+\frac{n\left({\text{EC}}_{\text{tr}}+\tau^{\prime }{\left(\text{Rw}\right)}^{\sigma^{\prime }}\right)}{N}\right],\\ A=2\;{\text{EC}}_{\text{tr}}+\tau e_{\text{tocj}}^{\sigma }+{\text{EC}}_{\text{ar}}. \end{array}$$

When the *R*th node passes through (1 − *a*) *T* rounds, the average energy consumption is

(10) $$\begin{array}{c} {\text{EC}}_{2}\left(\text{Rw}\right)=\left(1-a\right)T\left\{A+\frac{n}{N}\left[{\text{EC}}_{\text{tr}}+\tau^{\prime }w^{\sigma^{\prime }}+\frac{\mu_{n}^{2}-{\left(\text{Rw}\right)}^{2}}{{\left(\text{Rw}\right)}^{2}-{\left(\left(R-1\right)w\right)}^{2}}\left(2\;{\text{EC}}_{2}+\tau^{\prime }w^{\sigma^{\prime }}\right)\right]\right\}. \end{array}$$

The total energy consumption is

(11) $$\begin{array}{c} {\text{EC}}_{\text{Sum}}\left(\text{Rw}\right)={\text{EC}}_{1}\left(\text{Rw}\right)+{\text{EC}}_{2}\left(\text{Rw}\right). \end{array}$$

The expressions of the single-hop model and the multihop model are

(12) $$\begin{array}{c} {\text{EC}}_{d}=A+\frac{n\left({\text{EC}}_{\text{tr}}+\tau^{\prime }w^{\sigma^{\prime }}\right)}{N}, \end{array}$$

(13) $$\begin{array}{c} {\text{EC}}_{m}=A+\frac{n\left({\text{EC}}_{\text{tr}}+\tau^{\prime }w^{\sigma^{\prime }}\right)}{N}+\left(\frac{\mu_{n}^{2}-1}{w^{2}}\left(2\;{\text{EC}}_{\text{tr}}+\tau^{\prime }w^{\sigma^{\prime }}\right)\right). \end{array}$$

When Rw is *μ*_*n*_, the multihop expression is the same as formula (11), and the single-hop expression is

(14) $$\begin{array}{c} {\text{EC}}_{q}=A+\frac{n\left({\text{EC}}_{\text{tr}}+\tau^{\prime }\mu^{\sigma }\right)}{N}. \end{array}$$

The total energy consumption of the network in the hybrid routing mode is

(15) $$\begin{array}{c} {\text{EC}}_{\min}=\max\left\{E_{0}\left(R\right),E_{0}\left(\mu_{n}\right)\right\}. \end{array}$$

In 2002, the WSN network extended to the concept of a somatosensory network, namely, BSN. According to the low energy consumption and real-time characteristics of wireless networks, BSN networks can monitor the condition of their wearers in real time by installing certain sensor components. The ideal mobile health detection system should be portable, combined with multiple sensors, give real-time feedback, and provide wireless data communication to achieve online data evaluation. Researchers use infrared, electromagnetic, electronic, and biochemical technologies to develop a series of systems that can automatically monitor and identify unnatural parameters, such as body temperature, heart rate, ECG, blood pressure, and blood oxygen, and transmit signals through wireless communication and networks [15].

For example, some direct contact skin sensors can form an elastic sensor with air permeability with the help of some silica gel or expanded fibers. This sensor can perform skin manipulation and measurement through the skin. The system diagram of WSN for real-time monitoring of human health is shown in Figure 6. The user's relevant detection data are stored on the cloud database platform, and real-time data analysis is performed. The report sheet is returned to the user's application platform, and the user can judge the health status based on the relevant index data.

## 4. Experimental Research on the Detection Method of Human Body Nutrient Composition

Body composition refers to the body's total water content, blood sugar content, intracellular and extracellular fluid, vitamin content, fat mass and nonfat mass, and other parameters. It can reflect the nutritional status and fluid balance of the human body and comprehensively reflect a person's physical fitness level. The main body composition analysis methods used up to now are the skinfold method, body density method (such as the underwater weighing method and air displacement method), nuclear magnetic resonance imaging method, bioelectrical impedance analysis method, etc. They all have different advantages and disadvantages [16]. Among them, the skinfold method is economical but not very accurate; the human body density method uses a complicated device; the MRI method has radiation and is expensive and the portability is not high.

### 4.1. Human Body Composition Based on the Principle of Bioelectrical Impedance

The basic principle of the bioelectrical resistance analysis method is that the biological tissue contains many cells, and the liquid between the cells can be regarded as an electrolyte. When an electric current is applied through biological tissue, the resistance of the extracellular fluid and the intracellular fluid can be measured. The BIA method uses statistics as a tool. By studying the correlation between the impedance values obtained at different frequencies of the corresponding parts of the human body and some body composition parameters and combining the body weight, age, and gender parameters, the corresponding human body nutrition composition model formulas are established. Compared with other methods, the bioelectrical impedance analysis method has the following characteristics: one is a high accuracy, and this method is highly controllable and can model different human bodies; the second is easy to operate and relatively real time; the third is that the test indicators are more comprehensive, and numerous component data can be calculated. At present, some composition analysis equipment products are already on the market. The more typical one is the Inbody series from Biospace Corporation of South Korea. The main products are shown in Table 1 [17]. The main shortcomings of these instruments are the use of single-frequency measurement technology and the lack of phase detection. At the same time, the price is relatively expensive, so popularization and promotion are not used. Therefore, so far, the multifrequency measurement methods used at home and abroad have not fully realized impedance spectrum measurement. Most instruments only measure the impedance of the human body at certain frequency points.

Based on the *m*-sequence impedance spectroscopy measurement, the *m*-sequence can be better immune to interference signals. The autocorrelation function has special properties, and taking the 5-order *m*-sequence as an example, *N* is 31. The time-domain waveform, autocorrelation, and power spectrogram are shown in Figure 7.

The BIA human body structure analysis system designed in this document includes the upper computer position measurement, electrode circuit, and impedance circuit. The upper computer is responsible for running the programme, and the data returned to the platform are the interactive cloud between humans and computers that controls the analysis and display of the data to the user. The measuring circuit is responsible for measuring the weight of the human body, and the impedance measuring circuit is suitable for the safe current of the measured person. The electrode circuit is responsible for measuring the voltage of different parts of the human body and completing the data collection work. It calculates the impedance value of the human body and transmits it to the upper computer. The system software includes data analysis, time management, network management, and storage management [18, 19].

The interference control capability of the system can be tested by the noise signal ratio index. During the measurement, a current is injected from the left output pole and flows out from the right output pole. The maximum value of the current is 500,000 Hz, the number of measurements is 500 times, the number of sampling cycles is denoted by *M*, and the number of points used is denoted by *N*. Figures 8(a) and 8(b), respectively, show the noise signal ratio during different sampling periods and the noise signal ratio under different sampling frequencies. The actual sampling frequency set in this experiment is 25 MHz, and the sampling period number setting range is greater than 32. Therefore, when the constant current frequency is 1 MHz, the signal-to-noise ratio can continue to be greater than a critical value, and the anti-interference performance is good.

To measure the relative accuracy of the system, we set the current output frequency to 1 kHz during the test. The current output power is 0.5 mm, the resistance frame is used as the test object, and the resistance value ranges from 10 to 1000 ohms. It can be seen from the resistance measurement results of each channel that the measurement results of each channel are basically the same. The influence between different channels can be ignored, and the error is basically kept at about 2%. It tests the error under different signal output frequencies, and the results are shown in Table 2. The result shows that the higher the frequency, the greater the error, which reaches 18.6% at 1 MHz. The reason is that what the system measures is the impedance value, and the influence of distributed capacitance further increases the measurement error.

The human nutrient composition analyzer designed in this experiment and the seca mBCA-515 human nutrient composition analysis were used to test the nutrient composition of the test subjects. The subject was female, age 26, height 168 cm, and weight 60.6 kg. It compares the measurement results of the two instruments, and the comparison results are shown in Table 3. It can be seen from the data comparison results that, except for a few data with floating differences, most of the parameter values are consistent. This shows that the measurement results of the human nutrient composition analysis instrument designed in this paper are more accurate and can be used for human training and health monitoring.

### 4.2. Body Surface Sweat Electrochemical Sensor Wearable Portable Human Nutrition

Compared with other chemical detection technologies, electrochemical detection methods have the advantages of high sensitivity, high selectivity, low response time, and easy implementation of wearable designs. In recent years, various electrochemical sensing technologies have been used for wearable sweat analysis. One application area of the wearable sweat sensor is the health tracking and health monitoring of athletes in high-performance sports.

In high-intensity exercise and disease diagnosis, sweat biomarkers related to the physiological processes of the human body are usually the main objects to be detected. For example, these markers include electrolytes in human sweat (such as Na^+^, K^+^, Cl^−^, Mg^2+^, and Ca^2+^), metabolites (lactic acid, glucose), and micronutrients (such as iron, zinc, and tryptophan).

Sodium is one of the most important electrolytes in human sweat, and it is essential for the regulation of osmotic pressure, water balance, and pH. Sodium is an important biomarker for judging electrolyte imbalance, especially when the athletes perform a long-term exercise or are exposed to hot and humid environments. Sodium and chloride levels are also indicators of whether athletes are dehydrated during training, and ammonia content is related to extreme fatigue. Obtaining the physiological hydration level in real time will help to properly manage the electrolyte concentration. Lactic acid is usually produced during exercise, and the increase in lactic acid content in sweat is related to the transition from aerobic metabolism to anaerobic metabolism.

This experiment mainly takes sodium ion and potassium ion, the two ions with the highest content and the most obvious change in sweat, as the main test targets. It has prepared sodium and potassium all-solid-state ion-selective sensors. Sensors suitable for body surface sweat analysis must meet the characteristics of small system, light weight, flexibility, and high stability. The all-solid-state ion sensor can solve the difficulty of ion detection in the in situ analysis of body surface sweat. The experiments in this section are conducted on the prepared sensor electrodes to verify the performance of the prepared ion-selective electrodes.

#### 4.2.1. Stability Test

In actual physical training, the monitoring process of human nutrition is continuous dynamic sweat analysis. The sensor needs to work continuously, so the continuous stability requirements of the sensor are higher. In this study, the sodium ion- and potassium ion-selective electrodes are tested and analyzed for a long time, and the sensor is placed in a constant sample liquid for the experiment.

Figure 9 shows the long-term stability analysis results of sodium and potassium ions. In the experiment, let the sensor measure and record the electric potential in a 7 mM NaCl solution and then increase it to 14 mM. The curve rises clearly and continues to measure for several hours, and we find that it basically maintains the content in the stable range. The test result of potassium ion is shown in Figure 9(b), and the result is similar to that of sodium ion. It first detects the potential in a 0.8 mM standard KCl solution, then increases the concentration to 7 mM, and then performs long-term detection, and the curve remains stable. The fluctuation of the curve may be due to the formation of a thin water layer between the sensing film and the electrode surface, which affects the electrode potential. The test result shows that the selective electrode has a long-term stable detection ability, which can meet the long-term sweat detection and analysis needs.

#### 4.2.2. Sports Training Results

The physical test was performed on an indoor spinning bike, and the test watch was installed on the tester's right wrist. The ion-selective electrode is fixed to the 3D-PMD with double-sided tape and is connected to the smart watch through a plug-in connector. Before wearing the sensor, the wipe contacted the skin with a medical alcohol cotton pad to remove the surface oil. The subject was a male, aged 24, weighing 63 kg, and height of 172 cm. The test subjects pedaled indoors on a spinning bike to stimulate perspiration, and the test time was 50 minutes. When the test subject has a lot of perspiration, it is measured and the smart watch records it in real time.  Figure 10 shows the tester's real-time test data. The potassium ion concentration change is represented by a red line, and the sodium ion concentration change is represented by a green line.

At the beginning of the exercise, the tester had a small amount of sweat. Therefore, the start time of the data test was after 450 s. During exercise, the sodium ion concentration in sweat is related to the perspiration rate, which can reflect the size of the perspiration rate. It can be seen from the curve in the figure that the sodium ion level of the tester has a rising trend during physical training, from 43 mM to 58 mM. Potassium ions show a downward trend after a lot of perspiration; the trend gradually becomes smaller and finally stays at a stable level. The concentration of potassium ions and sodium ions can predict muscle activity and can calculate the content of various nutrients in the human body through models.

#### 4.2.3. Human Body Nutrition Based on Sweat Fluid Sensory Network on the Body Surface

Taking the real-time monitoring of glucose content as an example, 15 minutes before the start of the test process, each experimenter took honey water to simulate the sweat glucose level after a meal. It explains the large glucose concentration changes through exercise consumption. The electrochemical test is not performed ten minutes before the test, and it is only used for preperspiration. Then, perform half an hour of aerobic exercise for continuous perspiration, and then, take a ten-minute rest. The athlete's limbs remain still, the body returns to a peaceful state of metabolism, and the change in glucose concentration at this time is recorded. The test data of the tester, that is, the change curve of glucose concentration, is shown in Figure 11. The glucose concentration showed an obvious downward trend from a high level to a continuous decline. In the subsequent peaceful rest period, there is a certain upward trend. The tester's sweat glucose concentration was maintained at around 0.5 mM, but it was different from the glucose concentration level. It is higher than the glucose concentration, which may be the difference in the process of glucose diffusion and secretion from the blood to the surrounding tissue fluid and sweat glands, resulting in a different ratio of sweat glucose to blood sugar.

## 5. Discussion

The main research direction of the study is the real-time detection of body nutrition in sports training. The main technical and theoretical support is cloud computing technology and somatosensory network technology, which collect data in sports training. Cloud computing technology can analyze and process the data returned by the somatosensory network and generate a nutrition report to the trainer. This study first summarizes the relevant technical principles. The introduction of cloud computing content mainly includes an introduction to the basic content of cloud computing, cloud computing characteristics and logical structure, and cloud computing task allocation plan. In the introduction to the related principles of the somatosensory network, the main content revolves around the development background of the somatosensory network, technical principles, node transmission schemes, and wearable device models based on the somatosensory network. The study subsequently conducted performance experiments and results in comparison experiments on the real-time monitoring method of human nutrition in the process of sports training. This section is mainly composed of two sections of experiments. One section is an analysis experiment of human nutrition based on the principle of human electrical impedance. It mainly introduces the principle of the method, designs a body composition analysis system, and conducts a performance test of the system with the signal-to-noise ratio and error rate indicators. The results show that the performance of the system designed in this experiment is relatively stable, the error value is small, and all are within the acceptable range. After that, the measurement results of this system and the mBCA-515 body composition analyzer were compared, and the results showed that the measurement results of the system designed in this study were basically consistent with the measurement results of the mBCA-515 instrument. The second part of the experiment is the analysis of wearable human nutrition based on the electrochemical sensor of body surface sweat. In this experiment, the stability of the sensor system was tested. The results show that the selective electrode of the sensor has a long-term stable monitoring capability. Secondly, the experiment conducted a physical training test with sodium ions and potassium ions as the main detection targets and then conducted a human glucose concentration change test with the change of glucose concentration during physical training as the test purpose.

## 6. Conclusions

BIA technology has been widely used in human health detection, and sweat detection has now become a research subject of widespread concern. This study has mainly studied these two technologies, and there has been some progress in the experiment. However, there are still many shortcomings. For example, the nonexercise sweat detection may not be real time and accurate, and in the case analysis, there is no detection and analysis of multiple nutrients. In the field of sports health, it is necessary to fix sensors on the moving limbs. Therefore, the future prospect should be to improve the antimotion interference in the somatosensory network. For BIA technology, its research cost is relatively high, its size cannot meet the portability requirements, and it is not conducive to technology promotion and application.

## Figures and Tables

**Figure 1:** Cloud computing architecture model.

**Figure 2:** Cloud computing service characteristics.

**Figure 3:** Cloud computing logical structure.

**Figure 4:** Wireless sensor network structure.

**Figure 5:** Routing protocol structure.

**Figure 6:** Schematic diagram of real-time human body monitoring in WSN.

**Figure 7:** *m*-sequence analysis.

**Figure 8:** The signal-to-noise ratio of the number of sampling points under different sampling periods and sampling frequencies.

**Figure 9:** Stability results are measured over time.

**Figure 10:** Real-time trend chart of a smart wearable device sports training test. (a) Potassium ion. (b) Sodium ion.

**Figure 11:** Tester's glucose concentration curve.

**Table 1:** Biospace-inbody products.

Model	Measuring range (kHz)
Inbody-720	1,5,50,250,500
Inbody-220	20,100
Inbody 3.0	5,50,250,500

**Table 2:** Impedance frequency change.

Frequency (kHz)	Error (%)
1	2
5	1
10	−0.2
25	−0.8
50	−1
100	−2.3
250	−7.3
500	−12.2
1000	−17.6

**Table 3:** Comparison of measurement results for human nutrition.

Nutritional ingredient	mBCA-515	This experimental equipment
Total moisture (l)	34.2	34.1
Extracellular fluid (L)	12.8	12.6
Intracellular fluid (L)	21.6	21.7
Body fat (kg)	16.3	16
Fat-free body weight (kg)	44	43.5
Muscle weight (kg)	36.5	35.8
Protein (kg)	37.9	38.2
Inorganic salts (kg)	3.4	3.4

## Data Availability

The data that support the findings of this study are available from the corresponding author upon reasonable request.

## References

[1] Wei Z., Liu H., Wang W., Chen H., Ren C. (2019). Carbon dots as fluorescent/colorimetric probes for real-time detection of hypochlorite and ascorbic acid in cells and body fluid. *Analytical Chemistry*.

[2] Souza Ribeiro A., Bianchini D. (2017). The deployment of systems in cloud computing environment: a methodology to select and prioritize projects. *IEEE Latin America Transactions*.

[3] Deng R., Lu R., Lai C., Luan T. H., Liang H. (2017). Optimal workload allocation in fog-cloud computing toward balanced delay and power consumption. *IEEE Internet of Things Journal*.

[4] Abdel-Basset M., Mohamed M., Chang V. (2018). NMCDA: a framework for evaluating cloud computing services. *Future Generation Computer Systems*.

[5] Hirai T., Masuyyama H., Kasahara S., Takahashi Y. (2017). Performance analysis of large-scale parallel-distributed processing with backup tasks for cloud computing. *Journal of Industrial and Management Optimization*.

[6] Wennberg R., El-Rahimy Y., Shampur N., Dominguez L. G. (2017). Post-concussion abnormalities in the m60 somatosensory evoked field recorded by magnetoencephalography. *British Journal of Sports Medicine*.

[7] Botta M., Cancelliere R., Ghignone L., Tango F., Gallinari P., Luison C. (2019). Real-time detection of driver distraction: random projections for pseudo-inversion-based neural training. *Knowledge and Information Systems*.

[8] Farhan I. A., Al-Bakri J. (2019). Detection of a real time remote sensing indices and soil moisture for drought monitoring and assessment in Jordan. *Open Journal of Geology*.

[9] More P., Mishra P. (2020). Enhanced-PCA based dimensionality reduction and feature selection for real-time network threat detection. *Engineering, Technology & Applied Science Research*.

[10] Suryanarayana G., Chandran K., Khalaf O. I., Alotaibi Y., Alsufyani A., Alghamdi S. A. (2021). Accurate magnetic resonance image super-resolution using deep networks and Gaussian filtering in the stationary wavelet domain. *IEEE Access*.

[11] Shi C., Ning X., Sun Z., Kang C., Ma G. (2018). Quantitative risk assessment of distribution network based on real-time health index of equipment. *Gaodianya Jishu/High Voltage Engineering*.

[12] Ren Q.-Q., Wu J., Zhang W.-C. (2017). Real-time in vitro detection of cellular H_2_O_2_ under camptothecin stress using horseradish peroxidase, ionic liquid, and carbon nanotube-modified carbon fiber ultramicroelectrode. *Sensors and Actuators B: Chemical*.

[13] Shin M.-O., Oh G.-M., Kim S.-W., Seo S.-W. (2017). Real-time and accurate segmentation of 3-D point clouds based on Gaussian process regression. *IEEE Transactions on Intelligent Transportation Systems*.

[14] Kim M. G., Ko H., Pan S. B. (2019). A study on user recognition using 2d ecg based on ensemble of deep convolutional neural networks. *Journal of Ambient Intelligence and Humanized Computing*.

[15] Khan N. A., Khalaf O. I., Romero C. A. T., Sulaiman M., Bakar M. A. (2021). Application of euler neural networks with soft computing paradigm to solve nonlinear problems arising in heat transfer. *Entropy*.

[16] Vijayan V., Elizabeth S. (2019). Real time detection system of driver drowsiness based on representation learning using deep neural networks. *Journal of Intelligent and Fuzzy Systems*.

[17] Liu W. (2021). Real-time obstacle detection based on image semantic segmentation and fusion network. *Traitement du Signal*.

[18] Li J., Su Z., Geng J., Yin Y. (2018). Real-time detection of steel strip surface defects based on improved YOLO detection network. *IFAC-PapersOnLine*.

[19] Li G., Wang Q., Zuo C. (2021). Emergency lane vehicle detection and classification method based on logistic regression and a deep convolutional network. *Neural Computing & Applications*.

